RETRACTED

# Machine Learning-Based Automated Diagnostic Systems Developed for Heart Failure Prediction Using Different Types of Data Modalities: A Systematic Review and Future Directions

**DOI:** 10.1155/2022/9288452

**Published:** 2022-02-03

**Authors:** Ashir Javeed, Shafqat Ullah Khan, Liaqat Ali, Sardar Ali, Yakubu Imrana, Atiqur Rahman

**Affiliations:** ^1^Aging Research Center, Karolinska Institutet, Sweden; ^2^Department of Electrical Engineering, University of Science and Technology Bannu, Pakistan; ^3^Department of Electronics, University of Buner, Buner, Pakistan; ^4^School of Engineering and Applied Sciences, Isra University Islamabad Campus, Pakistan; ^5^School of Engineering, University of Development Studies, Tamale, Ghana; ^6^School of Computer Science and Engineering, University of Electronic Science and Technology of China (UESTC), Chengdu, China; ^7^Department of Computer Science, University of Science and Technology Bannu, Pakistan

## Abstract

One of the leading causes of deaths around the globe is heart disease. Heart is an organ that is responsible for the supply of blood to each part of the body. Coronary artery disease (CAD) and chronic heart failure (CHF) often lead to heart attack. Traditional medical procedures (angiography) for the diagnosis of heart disease have higher cost as well as serious health concerns. Therefore, researchers have developed various automated diagnostic systems based on machine learning (ML) and data mining techniques. ML-based automated diagnostic systems provide an affordable, efficient, and reliable solutions for heart disease detection. Various ML, data mining methods, and data modalities have been utilized in the past. Many previous review papers have presented systematic reviews based on one type of data modality. This study, therefore, targets systematic review of automated diagnosis for heart disease prediction based on different types of modalities, i.e., clinical feature-based data modality, images, and ECG. Moreover, this paper critically evaluates the previous methods and presents the limitations in these methods. Finally, the article provides some future research directions in the domain of automated heart disease detection based on machine learning and multiple of data modalities.

## 1. Introduction

A variety of conditions that affect the normal working of the heart are known as heart diseases. Heart diseases are classified into heart failure (HF), CAD, vessel disease, heart rhythm problems, and many more. Heart disease, also referred to as cardio vascular disease (CVD), defines the condition where the blood vessels are narrowed or blocked leading to a heart attack (myocardial infarction) and chest pain (angina). Symptoms of heart disease include chest pressure, chest discomfort (angina), shortness of breath, abnormal heartbeats, and heart defects [1]. HF is a chronic disease that affects the heart chambers. Cardiovascular disease abrupts the normal working of the heart that pumps sufficient amount of blood in the human body, without boosting the intracardiac pressure. As the heart becomes unable to pump sufficient blood to the rest of the body, the kidney reacts by inducing the body to retain fluid which results in lung congestion and swelling in the arms and legs. CHF is an expeditious healthcare problem [2] of the modern world, and 26 million adults around the globe are suffering from congestive heart failure [3]. Approximately 17.9 million patients with cardiovascular disease die every year that is 31% of the overall deaths around the world [4].

RETRACTED

Heart failure has many risk factors such as gender, family history, and increased age, which are classified into uncontrolled risk factors, while high cholesterol, smoking, high blood pressure, and obesity are classified into controllable risk factors [5]. To understand the HF, we explore and overview the most common types of heart failure diseases for better problem awareness. Herein, Figure 1 depicts the four chambers of the heart that are responsible for blood pumping.

In recent times, a large amount of data on patients has been generated in the healthcare sector. However, researchers and practitioners are not efficiently using this data for effective diagnosis of the disease. The healthcare sector is facing major challenges in quality of service (QoS) which ensures correct and timely diagnosis of disease that results in competent treatment of the patients. Impaired diagnosis leads to detrimental results which are not acceptable [7].

### 1.1. Major Types of Heart Diseases

#### 1.1.1. Coronary Artery Disease (CAD)

CAD is a heart disease which commonly occurs as result of the build of fatty deposits (plaque) inside the arteries responsible for supplying blood to the heart muscles. The obstruction in the arteries reduces blood flow to heart muscles which results in the impairment of the heart functions. This phenomenon is known as myocardial ischemia. The partial or complete blockage of arteries results in inevitable damage done to the heart also known as a heart attack. The human heart has four chambers that are divided into upper receiving chamber (right and left atria) and lower pumping chambers (right and left ventricle (LV)). The right atrium is responsible for gathering deoxygenated blood, and the right ventricle pumps the deoxygenated blood to the lungs for oxygenation process. Oxygenated blood from the lungs enters into the left atrium and is then transferred to all parts of the body through LV. The size and function of the LV chamber make it the most efficient responsible part of the heart. As such, the major reason for heart failure is due to damage of the LV chamber. Echocardiography helps in detecting CAD by examining or monitoring the heart for the evolution of CAD and wall motion abnormalities that begin to arise [8]. CAD can be diagnosed through LV measurement and wall motion scoring. Therefore, monitoring of LV is essential to avoid protracted damages that will affect size, shape, and function of the LV. Echocardiography is an imaging method that captures different cardiac views, structure, and their movement from ultrasound videos. Heart functional and morphological assessment is done to diagnose the cardiac disease through echocardiography [9]. Furthermore, echocardiography is also utilized for quantitative analysis of the LV ejection fraction and cardiac output [10].

RETRACTED

#### 1.1.2. Congestive Heart Failure (CHF)

Congestive heart failure also known as chronic heart failure is a condition whereby the heart fails to pump a sufficient amount of blood to the body to meet oxygen demand [11]. CHF is a chronic disease that affects the heart muscles. There are various risk factors behind CHF but the most common risk factors consist of high blood pressure, old age, obesity, and diabetes. Congestive heart failure is more common in men as compared to women. The term heart failure does not refer to the complete cease of the heart, but it actually diminishes the normal functionality of the heart as compared to a healthy person [12]. Heart failure means the body tissues are not getting enough blood and oxygen as needed for normal function. Systolic and diastolic are the two types of heart failures. In systolic heart failure, the pumping action of the heart is decreased. To test the systolic heart failure, a typical clinical test ejection fraction (EF) is done. The ejection fraction is measured as the amount of blood ejected out from the left ventricle (LV) divided by the maximum amount of blood remains in the left ventricle (LV) at the end of diastole. For a normal person, the value of ejection fraction is more than 55%, while for diastolic heart failure, the threshold value of ejection fraction is below 55%. In diastolic heart failure, the heart contracts normally but rigid and inflexible while it is relaxing and being filled with blood. Due to the stiffness of the heart, it is unable to be properly filled with blood to push back into the lungs which causes or leads to heart failure. The ejection fraction in diastolic heart failure is normal or hike.

RETRACTED

#### 1.1.3. Abnormal Heart Rhythms

Abnormal heart rhythms, also known as arrhythmias, are a condition whereby the heart beats too slow/too fast or irregularly due to a problem in the heart electrical system. The electrical system provides the heart with a clue of when to beat and supply blood to each part of the body [13]. Palpitations, tiredness, losing consciousness, dizziness, and breathlessness are the most common symptoms of an abnormal heart rhythm. The symptoms of heart failure are arduous to notice; therefore, it is also known as the silent killer. Doctors recommend various medical tests [14] for the diagnosis of heart failure, such as echocardiogram, where blood flow through the heart is monitored with the help of ultrasound waves. Electrocardiogram (ECG) is another way to diagnose heart problems related to the heart's rhythm. Holter monitoring is a portable device used to record continuous ECG data of the patient. Cardio computerized tomography (CT) scans provide the facility of an X-ray cross-sectional view of the patient's heart, to detect heart failure. Cardiac magnetic resonance imaging (MRI) helps to generate an image of the heart and tissues of the heart through the use of powerful magnets and radio waves.

We have studied three major types of heart diseases for which researcher has proposed ML-based automated diagnosis systems, but Figure 2 presents the detail view of the various heart diseases.

### 1.2. Rationale and Aim of the Study

Previous studies that reviewed automated methods for heart diseases mainly targeted one specific type of data modality. Moreover, those studies lacked highlighting the limitations in the previously developed automated methods for heart disease prediction. Hence, we provide a systematic review of automated diagnostic systems developed for heart disease prediction based on three commonly used data modalities which are images, ECG, and clinical feature-based data modalities as shown in Figure 3. Moreover, we discuss the development of image-based, ECG-based, and data mining-based diagnostic systems that exploit deep learning and ML algorithms for the automated diagnosis of heart diseases such as CAD, HF, CHF, and CVD. All the computer-aided detection systems based on ECG, images, and clinical feature-based data techniques have four key steps: preprocessing of data, features extraction, significant feature selection, and classification. Finally, we explore the potential issues in the diagnostic systems based on the images, ECG, and clinical feature-based data modality for heart disease detection and propose solutions. To meet this objective, data is gathered from various databases and sources like ScienceDirect, PubMed, IEEE Xplore Digital Library, Springer, Hindawi, Plos, and Google Scholar based on the keywords: automated heart disease prediction or detection, ML-based detection of CHF, prediction of heart failure, coronary disease detection, data mining, and CVD. The literature used in this study was selected on the basis of a particular criteria as given:

- Only CAD, HF, CVD, and CHF are targeted in this study
- The articles published from 1995 to 2021
- Those papers were considered that employed ML techniques for the diagnosis of the heart diseases
- The articles published in the English language are targeted in this study
- Articles that used different types of data modalities like ECG, images, and clinical features for automated detection of heart diseases were considered
- The research articles that made use of publicly available datasets and electronic health records

RETRACTED

## 2. Machine Learning for Heart Disease Prediction

Recently, large number of diagnostic systems have been developed for automated diagnosis of different diseases like Parkinson's disease [15–19], hepatitis [20], carcinoma [21], lung cancer [22], and mortality prediction systems [23, 24] using machine learning, deep learning [25], data mining [26], and optimization methods [27–30]. Heart disease detection through machine learning is not an exception, and recently, numerous approaches have also been successfully implemented on various datasets for automated heart disease detection [31–37]. The proposed algorithms have validated the efficient detection and prediction of heart failure. This study comprehensively reviews the ML approaches for HF prediction and detection based on three modalities (images, ECG, clinical features). This study provides the following key objects based on explicit analysis of the works that have been published in last 26 years:

- The proposed ML techniques on the basis of the modality used (such as images, ECG, clinical feature-based data), their benefits, and weaknesses
- The dataset properties according to modalities
- Performance measurement of the ML algorithms in terms of different evaluation metrics, namely, accuracy (ACC), specificity (Spec), and sensitivity (Sen)
- Comparative analysis of ML techniques based on a specific data modality

The results of this study present the best modality more suitable for the prediction or detection of HF through ML approaches. It also assists researchers and physicians to improve the quality of heart disease diagnosis. The comparative analysis in this study helps to identify the effectiveness and weaknesses of previously proposed ML techniques for the diagnosis of heart disease and also suggests challenges in future works for accurate, reliable, and cost effective development of automated diagnosis system.  Figure 4 provides an overview procedure for automated diagnostic system.

RETRACTED

### 2.1. Article Selection

The articles selection procedure was based on the three modalities (clinical feature-based data, images, ECG) for heart disease diagnosis. We collected 105 research articles on CHF and CAD detection from various publishers such as IEEE, MDPI, Springer, Elsevier, Hindawi, and PubMed based on the keywords CAD, HF, CVD, ML, deep learning, neural networks, etc. 35 articles were selected for each modality. Researchers around the globe have been working on ML-based heart disease detection system since 1992 [38] but the number of research papers in this domain as of 2014 was very limited. In recent years, researchers have developed a lot of CAD and HF detection systems based on ML. Therefore, the number of research papers in this field has seen a tremendous increase as depicted in Figure 5.

### 2.2. Datasets

This section describes the datasets that are considered in the selected research articles for experiments and performance evaluation of the developed automated diagnostic systems. A total number of 56 datasets are considered from the selected research articles. These datasets are collected from various organizations all over the world. Few datasets are publicly available while others are collected by researchers from different hospitals and healthcare organizations. We only listed those datasets that are used for diagnosis of HF, CVD, CHF, and CAD by using ML and data mining techniques. As our study is based on the three heart disease modalities, we therefore considered datasets based on these modalities. Thus, datasets differ in terms of samples and number of features.

Table 1 depicts the properties of datasets in terms of number of subjects, dataset features, missing values, etc. Based on the modalities (clinical feature-based data, images, ECG), the nature of the datasets is diverse. For instance, dataset IDs 01, 02, and 09 are used for patients' medical reports data (age, sex, chest pain type, resting blood pressure, etc.). The most famous dataset used in clinical feature-based data modality is UCI datasets, namely, Cleveland dataset, Hungarian dataset, Switzerland dataset, and Statlog dataset. UCI datasets consist of clinical features (age, serum cholesterol, exercise induced angina, etc.) that are used for automated diagnosis of HF through ML techniques. Other well-known datasets that belong to the clinical features modality are Z-Alizadeh Sani dataset and Extended Z-Alizadeh Sani dataset. Some datasets are based on ECG modality. ECG signals are used to record patients' medical data. ECG-based datasets are used by the researchers through ML and data mining approaches for the prediction and detection of the CVD and CHF disease. ECG signals are sampled to extract features from the signals. The extracted features are then used for training and testing purposes through ML models. Dataset IDs, 19, 20, 21, etc., are examples of the ECG datasets (MIT/Beth Israel Hospital (BIH), arrhythmia database, Physikalisch-Technische Bundesanstalt diagnostic ECG database). Image-based datasets consist of features that are extracted from the medical image data. ML approaches are deployed for extracting features from the images. Furthermore, models are trained and tested based on the features for automated diagnosis of the HF and CVD disease. Dataset IDs 30, 31, 32, etc., are instances of image based datasets (Cedars-Sinai Medical Center, Los Angeles CA and MCG data, Hospital Fernando Fonseca dataset). Moreover, Figure 6 depicts in detail the total number of samples in a given dataset along with total numbers of features for different datasets.

RETRACTED

## 3. Automated Heart Disease Detection Based on Different Modalities

### 3.1. ML-Based HF Diagnosis: Clinical Feature-Based Data Modality

In recent years, data mining and ML researchers have proposed different automated methods for heart disease detection based on clinical feature-based data modality [16, 17, 39]. For example, Verma et al. [40] developed a hybrid system for the prediction of CAD using noninvasive clinical data. Their hybrid system used correlation-based subset (CFS) selection and particle swam optimization (PSO) search technique to reduce the feature space from the dataset for better performance. A number of optimized feature subset are then input into the proposed model. The model is composed of multinomial logistic regression (MLR), multilayer perceptron (MLP), C4.5, and fuzzy unordered rule induction algorithm (FURIA). The proposed model is tested on the dataset of IGMC that has 26 features and 335 subjects. MLR achieved the highest accuracy of 88.4% while for benchmark dataset such as Cleveland heart disease, it obtained an accuracy of 90.28%. Shah et al. [41] proposed a method that extracted high impact features from the feature space by using probabilistic principal component analysis (PPCA). PPCA was used to extract the new feature vectors that helped to reduce the feature space. New feature vectors were selected by parallel analysis (PA). These reduced feature vectors were supplied to the radial basis function (RBF) kernel-based support vector machine (SVM). The RBF function performed the job classification into types, i.e., normal subject and heart patient. The proposed system achieved the accuracy of 91.30%, sensitivity of 100%, and specificity of 50%. Ali et al. proposed a novel method based on optimized and stacked support vectors machine and obtained 92.22% of HF prediction accuracy [42]. In another study, Ali et al. developed a hybrid system based on *χ*^2^ statistical model and deep neural network and further improved the HF prediction accuracy to 93.33% . In yet another study, Ali et al. highlighted the problem of overfitting to the testing data and proposed the development of mutually informed neural networks for better generalization of the decision support systems developed for HF prediction [43]. Dwivedi [44] evaluated the performance of the six ML methods on the data of StatLog heart disease dataset [6 King RD (1992) Statlog databases. Department of Statistics and Modelling Science, University of Strathclyde, Glasgow] for heart disease prediction. The performance of the ML techniques was evaluated through *k*-fold crossvalidation test. The highest accuracy of classification was reported in this study (85%) with sensitivity of 89% and specificity of 81% through logistic regression.

RETRACTED

An ML-based system was proposed by Guidi et al. [45] for the assistance of heart failure patient. Clinical decision support system (CDSS) has two major components for providing the assistance to heart patients. One of the component evaluates the severity of the HF while the other component predicts the HF. Additionally, CDSS also provides an interface for the comparison of various patient's follow-ups. The core of the CDSS was developed based on ML techniques such as SVM, NN, RF, and fuzzy-genetic rules. A supervised database was populated for ML techniques. The number of patients in the database was 90 with 136 records. The proposed CDSS was tested through the *K*-fold crossvalidation scheme. The prediction performance was reported with respect to the ML models as NN: 84.73%, SVM: 85.2%, fuzzy-genetic: 85.9%, CART: 87.6%, random forest: 85.6%, and severity performance given as NN: 77.8%, SVM: 80.3%, fuzzy-genetic: 69.9%, CART: 81.8%, and random forest: 83.3%.

Pawlovsky [46] designed an ensemble model using distance for KNN (*k* nearest neighbor) method for the diagnosis of heart disease. The proposed model was implemented by using three distances and five-distance configuration. A weight is also added at the base of the average accuracy that was calculated through KNN. The dataset used in this study was Cleveland, UCI dataset, and an average accuracy reported through the proposed system was 85%. Yu and Lee [47] proposed a system for CHF recognition based on heart rate variability through bispectrality analysis and genetic algorithms. Bispectrality analysis and genetic algorithm were used for the feature selection while SVM employed was a classifier. The proposed system obtained the accuracy of 98.79%.

RETRACTED

Wang et al. [48] proposed a deep ensemble model for the detection of CHF through short-term RR intervals and deep neural network. For the experiments, they selected five open-source databases, namely, BIDMC Congestive Heart Failure Database (BIDMC-CHF), MIT-BIH Normal Sinus Rhythm (NSR) database), Congestive Heart Failure RR Interval Database (CHF-RR), Normal Sinus Rhythm RR Interval database (NSR-RR), and Fantasia database (FD). To evaluate the proposed method, three RR segment length types (*N* = 500, 1000, and 2000) were used. Deep learning features were automatically extracted from the expert feature of RR intervals, a long/short-term memory-convolutional neural network-based. The proposed method achieved the accuracy of 99.85%, 99.41%, and 99.17% on *N* = 500, 1000, and 2000 length RRIs.

Methaila et al. [49] designed a heart disease prediction system based on data mining techniques. The proposed system used ML methods, i.e., decision tree, NB, and NN for the prediction of heart disease. An online dataset from the Cleveland Heart Disease database was utilized for the experiments. To reduce the feature dimension, apriori algorithm and frequent pattern mining using MAFIA were deployed. Significance weight calculation of the features was evaluated for better feature selection. Results from the proposed research suggest that decision tree outperformed the other ML techniques with accuracy of 99.62% while using 15 features.

Jan et al. [50] proposed an ensemble model based on multiple classifiers for better prediction accuracy of the heart disease. In this study, SVM, Naive Bayesian, linear regression, ANN, and random forest were combined to improve the prediction accuracy. An open source dataset from Cleveland and Hungarian CVD had been utilized for the experiments to evaluate the performance of the proposed model. The dataset had 76 features, but for the experiments, Jan et al. focused on 13 key features of the dataset that highly contributed to obtain the highest accuracy. *K*-fold crossvalidation (with *k* = 10) scheme was employed to validate the results of the proposed model. The proposed model obtained the accuracies according to classifiers as given, Naive Bayesian: 93.223%, ANN: 94.915%, SVM: 98.136%, and LR: 93.22%.

Pecchia et al. [61] developed a remote health monitoring system for the detection of heart failure. Data mining technique was employed with CART method and HRV for feature extraction. The proposed system achieved the accuracy of 96.39% and precision of 100.00%, respectively, for heart failure detection. In regards to severity assessment of HF, the achieved accuracy was 79.31%, and precision was 82.35%. A public dataset of Congestive Heart Failure RR Interval Database was utilized for the experiments. The total number of subjects in the dataset was 83 of which 54 were healthy and 29 were suffering from HF. Kurnar [62] proposed a method for heart disease detection using fuzzy resolution mechanism. The proposed method was based on the combination of ANN and fuzzy logic. The method is tested on an online open source dataset of heart disease from Cleveland. The proposed ANFIS model achieved the accuracy of 91.83%. All the experiments were done through MATLAB.

RETRACTED

Khumar et al. [82] proposed an ML-based method for the diagnosis of CVD. Dataset used in their work was collected from UCI, Cleveland, for testing the performance of the proposed model. Data cleaning techniques were employed for eliminating noise from the data. The processed data was input to the ML method for classification. The result reported from the proposed method obtained an accuracy of 86%.

Panicacci et al. [63] evaluated ML algorithms for identification of the heart failure patient. The dataset used for this study was collected from the Agenzia Regionale Sanit'a (ARS) in Florence, Tuscany, Italy. Panicacci et al. obtained the highest accuracy of 99.75% by random forest trained with SMOTE28 set. Latha et al. [64] investigated the ensemble classification method for improving the accuracy of weak algorithms through combination of multiple classifiers. The proposed method used dataset from the Cleveland heart disease dataset. The ensemble classification method of Latha et al. obtained an accuracy of 85.48%. Zikos et al. [65] conducted a Bayes study for the dynamic effect of comorbidities on hospital care for CHF patients. For this study, medical claimed data from centers for medicare and medicaid service (CMS) was collected. Bayesian scenario-based graphs and Bayes-networks were used to visualize the results.

Das et al. [5] developed a neural network ensemble model for effective diagnosis of heart disease. Their methodology used SAS base software 9.1.3 for heart disease detection. The neural network ensemble was the key element in their proposed method that developed new models from the posterior probabilities. The proposed model obtained the accuracy of 89.01% with 80.95% and 95.91% sensitivity and specificity, respectively. Mohan et al. [66] proposed a hybrid random forest with linear model (HRFLM) for CVD prediction. Their proposed model found the key features on which ML techniques provided improved accuracy for CVD. To test the effectiveness of the proposed model, an online open source dataset for Cleveland heart disease from UCI was collected. The accuracy achieved by HRFLM model was 88.7%.

RETRACTED

A hybrid neural network system based on ANN and FNN was proposed by Kahramanli and Allahverdi [67]. To validate the performance of the proposed model, an online line dataset from the ML repository was collected. The UCI heart disease dataset was employed for performance evaluation. The proposed system obtained an accuracy of 86.8%. Maji and Arora [68] presented a hybrid method based on ANN and decision tree for improved prediction of the heart disease. The UCI dataset is used to evaluate the effectiveness of the proposed model with WEKA tool. Tenfold crossvalidation testing is used to report the accuracy, sensitivity, and specificity of the proposed system. The system achieved the accuracy, sensitivity, and specificity of 78.14%, 78%, and 22.9%, respectively.

Polat et al. [69] proposed an artificial immune recognition system (AIRS) for heart disease diagnosis. Their proposed system used fuzzy weighted preprocessing method for extracting new features from the features space. The new features were input to the AIRS for prediction of the heart disease. The proposed system achieved an accuracy of 96.28% on an open source dataset of heart disease from UCI ML repository. To evaluate the performance of the proposed system, 10 *k*-fold crossvalidation testing was done. A comparative study of neural networks with traditional methods of medical diagnosis was done by Ster and Dobnikar [70]. In this study, five types of datasets were utilized for diagnosis of three kinds of diseases which were CAD, breast cancer, hepatitis, diabetes, and heart disease. The results of the study were obtained on default parameters. The highest accuracy achieved for heart disease by LDA was 84.5% and 59.7% for CVD by SNB.

Chen et al. [71] developed a CHF detection method through deep learning with RR intervals. Features from the dataset were extracted through the use of autoencoder. Extracted features were then supplied to deep neural network. The proposed system obtained an accuracy of 72.41% with sensitivity and specificity of 48.78% and 85.72%, respectively. Rajliwall et al. [73] proposed an ML-based CVD prediction model. A scalable algorithm named as the neuron network was presented which attained accurate results on fuzzy data. To evaluate the performance of the proposed model, two open source datasets were collected for the experiments. The best accuracy of 98.5% was obtained by random forest. Samuel et al. [74] proposed a model based on the fuzzy analytic hierarchy process (Fuzzy_AHP) technique that computed the global weight of the features for their individual contribution. Higher global weight features were supplied to the ANN classifier for prediction of heart failure. Cleveland dataset on heart disease from the UCI online repository was utilized for evaluating the performance of the proposed model. The proposed model obtained an accuracy of 91.10%.

RETRACTED

Venkatalakshmi and Shivsankar [75] developed a predictive model for the heart disease diagnosis. The proposed model was based on the Naive Bayes and decision tress. The dataset used for the experiments was heart disease dataset from UCI. Wake tool was utilized for the extraction of useful features from the dataset. The proposed model achieved an accuracy of 85.03% for Naive Bayes and 84.01% for decision tree. Maio et al. [76] developed a predictive model of hospital mortality for heart failure patients through improved random survival forest. A public dataset of MIMIC II clinical database which consisted of 8059 patients with 32 features was used for the experiments. The proposed system achieved the accuracy of 82.01%.

A computer-aided decision-making system based on hybrid neural network-genetic algorithm for heart disease detection was developed by Arabasadi et al. [34]. To evaluate the performance of the hybrid system, Z-Alizadeh Sani dataset was used for the experiments. 10-fold crossvalidation was used as performance measurement metric. The proposed system achieved an accuracy, sensitivity, and specificity of 93.85%, 97%, and 92%, respectively. A normalized technique was developed for the preprocessing of the data. A genetic algorithm along with particle swarm optimization was utilized for improving the performance. For performance evaluation of the proposed method, 10-fold crossvalidation was performed. A new optimization method N2Genetic optimizer was proposed in this study. Experimental results of the proposed method N2Genetic-nuSVM demonstrated that the proposed method achieved an accuracy of 93.08% and f1-score of 91.51%.

Laskshmi and Haritha [79] proposed a ML model using SVM and Naive Bayes. In this study, an online dataset from the Cleveland heart disease dataset was collected for the experiments purpose. The result of the proposed model was validated from the ROC chart, and reported accuracy was 84.87%. Javeed et al. [81] presented an intelligent learning system based on a random search algorithm and optimized random forest model for improved heart disease detection. For feature selection, random search algorithm was used by the proposed diagnostic system while the grid search algorithm was used for optimization. Experiments were performed using an online heart failure database, namely, Cleveland dataset. The proposed system used only 7 features for the detection of heart disease. The accuracy obtained by the newly proposed system was 93.33%.  Figure 7 presented the various ML models based on clinical feature-based data modality.

RETRACTED

### 3.2. ML-Based HF Diagnosis: Image Modality

Apart from the automated diagnostic systems based on clinical features, many researchers also exploited the use of imaging data modality for the development of automated methods for heart disease detection. For example, Nirsch et al., [83] proposed a deep learning classifier for the identification of heart failure patients based on whole slide images of H&E tissue. The gold-standard for the diagnosis of heart failure is an end myocardial biopsy (EMB) when the cause of the heart failure is not identifiable. The proposed method used the CNN for the detection of heart failure from H&E stained whole-slide images from a dataset collected from the university of Pennsylvania with 209 patients. To evaluate the performance of the proposed model, a 3 *k*-fold crossvalidation method was deployed, and the reported accuracy with sensitivity and specificity of the proposed method was 97.4%, 99%, and 94%, respectively.

Cetin et al. [84] developed a radiomic approach of computer-aided diagnosis through cardiac cine-MRI. To reduce the feature dimensionality, sequential forward feature selection (SFFS) algorithm was selected, while for the classification purpose, SVM classifier was used in the proposed model. To evaluate the performance of the proposed model, a dataset of 100 patients was collected from the university of the Hospital of Dijon (France), and crossvalidation metric was used for performance evaluation. Bai et al. [85] proposed a method for myocardial patient classification through shape and motion features. The proposed method used principal component analysis (PCA) for features selection of the shape features, whereas motion features helped to identify the wall motion and thickness of the wall. The performance of the proposed model was evaluated on the dataset of STACOM 2015 challenge. SVM was used for the classification which achieved a maximum accuracy of 97.5%.

Qazi et al. [86] proposed a spare linear classifier for the automated detection of heart abnormality. The proposed model was developed from linear fisher's discriminant (LFD). The dataset used in this study was collected from the St. Francis Heart Hospital in Roslyn, New York. This dataset consists of a total 200 subjects amongst which 141 cases were used for the training purpose, while 59 cases were marked for testing. The performance of the proposed model was valuated with other ML methods such as SVM, RVM, and LED. The accuracy achieved by the proposed model was 89.6%, which outperformed the other ML methods. Sanj and Kukar [87] studied the image processing and ML method for medical imaging. The proposed approach suggested that significant improvement could be achieved in automated diagnostic system by improving the posttest diagnostic probabilities, using multiresolution image parameterization and feature subset selection in conjunction with ML approaches. The proposed approached achieved an accuracy of 81.3% with PCA on ArTex/Ares parameters.

RETRACTED

Arsanjani et al. [88] proposed a method for earlier prediction of CVD through image features derived from SPECT (MPS) by a ML approach. For automatic feature selection, boosted ensemble ML algorithm (LogitBoost) was utilized for the prediction revascularization. To validate the effectiveness of the proposed model, tenfold crossvalidation scheme was adopted. The proposed model achieved an accuracy of 81% and was also tested through receiver operator characteristics (ROC) area under the curve. Udovychenko et al. [89] proposed a binary classification method for heart failure detection based on myocardial current density distribution maps. In this proposed method, KNN was utilized for the classification, while for performance validation of the proposed method, Matthews correlation coefficient (MCC) performance evaluation metric was selected. The proposed method reported an accuracy in the range of 80-88% with 70-95% sensitivity, 78-95% specificity, and 77-93% precision, respectively.

Berikol et al. [93] proposed a method for the diagnosis of the acute coronary syndrome through SVM. Laboratory tests and ECG data were used for the experiment. Data was collected and proved by the Mersin University Research and Training Hospital Ethics Committee for this study. The dataset consists of 228 patients image records. The proposed system based on SVM classifier obtained the accuracy, sensitivity, and specificity of 99.13%, 98.22%, and 100, respectively. Leader et al. [94] developed an approach for automatic characterization of plaque composition in carotid ultrasound using convolutional neural network. CNN was used to extract information from the medical images that helped in the identification of different plaque constituents. For this study, 90000 patches extracted from the dataset of images were obtained from the University Hospital Arnau de Vilanova, Lleida, Spain. To validate the performance of the proposed model, *k*−-fold crossvalidation scheme was adopted. The proposed approach obtained the accuracy of 90%.

Sundaresan et al. [95] proposed an automated characterization approach for the fetal heart through ultrasound images based on a fully convolutional neural network (FCN). FCN was trained on 10,000 random sample frames with 10 subjects and tested on 2178 frames with 2 subjects. ROC chart was used to validate the performance of the proposed approached. The classification error reported through the proposed model was 23.48%. Choi et al. [96] designed a model for early detection of heart failure from the onset by using recurrent neural network (RNN). The proposed model used gated recurrent units (GRUs) for the detection of relationship of time-stamped events. The dataset used for the experiments was collected from the Sutter Palo Alto Medical Foundation. The performance of the proposed model was evaluated against various ML models like SVM and KNN. The proposed model achieved the highest accuracy of 83.3% as compared to the other ML models SVM (74%) and KNN (73%).

RETRACTED

Mariachi et al. [98] proposed a framework for the detection of fetal presentation and the heartbeat through linear ultrasound video. The proposed framework classified frames into a 2D slice of the video. A conditional random field model was deployed for the regularized classification scores through temporal relationship between video frames. The kernelized linear dynamic model identified that heartbeat was detected in the frame sequence. For experiment purpose, a dataset of 323 predefined free-hand video was taken. The proposed framework reported a classification accuracy of 93.1% for the detection of a heartbeat.

Kurgan et al. [99] proposed a knowledge discovery method for automated cardiac SPECT diagnosis. A dataset of 267 patients consisting of SPECT images with 3000 2D images was used. A user friendly algorithm was designed for automated diagnosis. The proposed approach achieved an accuracy of 83.96%. Allsion et al. [104] proposed a model for detecting extensive CAD through artificial neural network for the modeling of stress single-photon emission computed on tomographic imaging. The dataset consisting of 109 patients of stress single-photon emission was collected for the experiments. The proposed model reported a sensitivity of 92%. Curiale et al. [106] proposed a method for automated myocardial segmentation through deep learning network in cardiac MRI. To evaluate the performance of the proposed method, Dice's coefficient and a mean squared error scheme are utilized. The proposed method achieved an accuracy 90%.

Moreno et al. [109] proposed a model for cardiac disease prediction through regional multiscale motion representation. The dataset was collected from the MICCAI challenge, Sunnybrook Cardiac Data (SCD) for the experiments. The SCD consist of 45 cine-MRI images. For classification of the heart disease, random forest algorithm (RAF) was employed. The performance of the proposed model was evaluated through two performance measurement metrics which are F1 score and the number of true positive from the total sample space. The proposed model obtained the average accuracy of 77.83% and F1 scored accuracy of 76.92%. Gulsun et al. [110] proposed a method for coronary centerline extraction via optimized flow paths along CNN path pruning. The proposed method automatically extracted the blood vessel centerlines. CNN is used as a classifier in the proposed method for removing extraneous paths. The proposed method was evaluated against 106 clinically annotated coronary arteries data. The proposed method achieved a specificity and sensitivity of 90% and 97%, respectively. Betancur et al. proposed a method of prognostic value of combined clinical and myocardial perfusion imaging data through ML. The predictive value of combined clinical information and myocardial perfusion single-photon emission was computed on tomography (SPECT) imaging (MPI) data based on ML for predicting the major adverse cardiac events. For the experiments, a total of 2619 patients' data were collected. The performance of the proposed model was evaluated through 10 *k*-fold crossvalidation. The accuracy achieved by the proposed model was 81%.

RETRACTED

Wolterink et al. proposed an automatic coronary calcium scoring in cardiac CT angiography through convolutional neural networks. The proposed method presented a pattern recognition method that helped to identify coronary artery calcium (CAC) in coronary computed tomography angiography (CCTA). The dataset consists of 50 patients which was used for the experiments based on five cardiovascular risk categories. CNN was deployed for the identification of the coronary artery calcium (CAC), and an accuracy of 95% was achieved by the method.  Figure 8 presented the performance various ML techniques based on image data modality.

### 3.3. ML-Based HF Diagnosis: ECG Modality

Similar to the clinical features and imaging modalities, numerous researchers also developed diagnostic systems based on ECG data modality for the detection of heart disease. For example, Zhao et al. [118] studied the simultaneous analysis of heart rate variability (HRV) and pulse transit time variability (PTTV) on healthy subjects and heart patients with the purpose of examining the improvement of HRV-based HF detection by using PTTV. For this objective, a data of 40 subjects through standard limb lead-II electrocardiogram (ECG) and radial artery pressure waveforms (RAPW) was collected. Moreover, SVM was deployed for the classification purpose along with probabilities generated from the distance distribution matrix- (DDM-) based CNN. The study demonstrated the accuracy, sensitivity, and specificity of 90%, 93%, and 88%, respectively. Sudarshan et al. [119] proposed a novel method for automated diagnosis of CHF based on dual tree complex wavelet transform and statistical features extraction from ECG signals. Dual tree complex wavelet transform (DTCWT) was performed on ECG segments for 2 seconds to obtain the six level coefficients. Features from the DTCWT were extracted through rank implementation using Bhattacharyya, entropy, minimum redundancy maximum relevance (mRMR), receiver-operating characteristics (ROC), Wilcoxon, *t*-test, and relief methods. For classification, ranked features were tested through *K*-nearest neighbor (KNN) and decision tress (DT). The proposed method reported the accuracy, specificity, and sensitivity of 99.86%, 99.94%, and 99.78%, respectively.

RETRACTED

Acharya et al. [120] proposed a model that automatically detected the CAD using various durations of ECG segments with CNN. For this study, a dataset of fantasia was collected from the Physionet database to evaluate the performance of the proposed model. ECG signal (lead II) from 40 healthy subjects (20 males, 20 females) and 7 CAD patients (1 male and 6 females) data was collected. The proposed method reported the accuracy, specificity, and sensitivity of 99.86%, 99.94%, and 99.78%, respectively. Chen et al. [121] proposed an early predictor of heart problems by using predictive analysis of ECG signals. The proposed method was based on a two-step predictive framework for ECG signal processing. A global classifier factor was employed to compare the abnormalities against a universal reference model. The proposed model obtained a classification accuracy of 96.6%.

Shen et al. [122] analyzed the ECG data for the risk prediction of CVD. ML techniques were employed for the improved risk evaluation of CVD through ECG. Their work investigated the detection of heart abnormality by using 3 one-class classification, predicting probabilities of normality, ischemia, hypertrophy, and arrhythmia through multiclass approach. One-class approach obtained the accuracy of 75.6% and an area-under-curve (AUC) of 83%. With a four-class approach, a classifier accuracy of 75.1% was achieved. Acharya et al. [123] designed an automated characterization of arrhythmias through nonlinear feature from tachycardia ECG beats. For classification, KNN and decision tree (DT) were employed. Open source datasets from MIT-BIH A-Fib Database, MIT-BIR arrhythmia database, and Creighton University VT Database were collected for acquiring the ECG signals. The proposed model achieved an accuracy of 96.3% with specificity and sensitivity of 84.1% and 99.3%, respectively. Mathews et al. [124] proposed a deep learning-based method for ventricular and superventricular heartbeat detection by using single-lead ECG classification. The proposed method was evaluated with data collected from the MIT-BIH database. Restricted Boltzmann machine (RBM) and deep belief network (DBN) were utilized to obtain an average identification accuracy of 93.63% for ventricular ectopic beat and supraventricular ectopic beats (95.57%) at a low sampling rate of 114 Hz.

RETRACTED

Adam et al. [125] proposed an automated characterization of CVD through relative wavelet nonlinear feature extraction of ECG signals. A novel discrete wavelet transform (DWT) method along with nonlinear features was used for automated characterization of CVD. Relative wavelet from four nonlinear features such as fuzzy entropy, sample entropy, signal energy, and fractal dimension was extracted from the DWT coefficients. Features were then supplied to sequential forward selection (SFS) algorithm to rank relief method. The proposed methodology achieved an accuracy, sensitivity, and specificity of 99.27%, 99.74%, and 98.08%, respectively, with KNN classifier using 15 features ranked by relief. Tang et al. [126] developed a system for accurate identification of the CAD through stacked CNN and long short-term memory management network from ECG signals. CNN was utilized to extract features from the dataset of ECG samples. The proposed method based on a deep learning technique successfully detected CAD from the ECG signals with a diagnostic accuracy of 99.85%.

Sharma et al. [127] proposed a novel automated diagnostic system for myocardial infraction through ECG signals, based on the optimal biorthogonal filter bank for classification. Physikalisch-Technische Bundesanstalt database was used to get the raw ECG signals. An optimal biorthogonal filter bank (FB) was employed for the ECG signal analysis. The ECG signal was decomposed into six sub bands (SBs) through a newly developed wavelet FB. For features extraction, fuzzy entropy, renyi entropy, and signal-fractal-dimension (SFD) were used to compute the six SBs. KNN was used for the classification problem based on the features obtained through SBs. The proposed system obtained an accuracy of 99.62% for raw data and 99.74% for clean data.

Pucer et al. [128] proposed a topological method for delineation and arrhythmic beat detection from unprocessed long-term ECG signals. The proposed approach was based on the subject, specific adaptation of the one-dimensional discrete Morse theory (ADMT). The ADMT technique was used for noise removal and detection of the characteristic waves of the subject ECG beats. The waves were labeled with the help of ADMT technique. A decision tree algorithm was used for classification based on the input labeled beats. The proposed system used MIT-BH dataset for the performance evaluation and a classification accuracy of 92.73%, sensitivity, and specificity of 73.35% and 96.70%, respectively, were reported. Huang et al. [129] proposed a vector cardiogram-based classification system for the myocardial infarction detection. For the experiments, an open source VCG dataset of PTB database from the Physionet was collected. The dataset consists of 448 VCG recording (80 healthy controls (HCs) and 369 MIs). For the features, selection FFS and BFS were employed. The proposed method used four classifiers (MLC, k-NN, GLM, and SVM) for the classification. The proposed system obtained an overall accuracy of 96.96% with 99.89% sensitivity and 92.51% specificity. Zhou et al. [130] designed a model for premature ventricular contraction detection from ambulatory ECG using recurrent neural networks (RNN). The proposed model tested with MIT-BIH arrhythmia database and the accuracy reported in range of 96%-99%.

RETRACTED

Sudarshan et al. [119] proposed a method for an automated diagnosis of CHF based on dual tree complex wavelet transform. From experiments, the coefficients were obtained through DTCWT implementation on ECG segments of 2 second duration to six levels. The statistical features were extracted and ranked by using Wilcoxon, *t*-test, relief methods, entropy, minimum redundancy maximum relevance (mRMR), receiver-operating characteristics (ROC), and Bhattacharyya. For automated diagnosis of the CHF, ranked features were classified through decision tree and KNN. The proposed method obtained an accuracy of 99.86%, with sensitivity and specificity of 99.78% and 99.94%, respectively. Diker et al. [132] proposed a new technique for heart disease detection through ECG signal classification, genetic algorithm, and wavelet kernel extreme learning machine. For the experiment, they utilized the Physikalisch-Technische Bundesanstalt Diagnostic ECG Dataset (PTBDB) from the Physionet Database. The critical points QRS complex, PR, QT, and ST from ECG signals were extracted through discrete wavelet transform (DWT) methods. Then, extreme learning machine (ELM) techniques were implemented on the ECG signals to find out the coefficients that were used in the wavelet kernel extreme ML. The proposed method achieved an accuracy of 95% along with sensitivity and specificity of 100% and 80%, respectively.

Acharya et al. [133] proposed a deep neural network based method for automated detection of the myocardial infraction through ECG signals. The dataset for the experiments was collected from the Physikalisch-Technische Bundesanstalt Diagnostic ECG Database (PTBDB) from Physionet. The proposed method was implemented without features extraction or feature selection method. The average accuracy of the proposed method using ECG beats with noise and without noise was 93.53% and 95.22%, respectively. Yao et al. [134] proposed a method based on the attention-based time-incremental convolutional neural network (ATI-CNN) for multiclass arrhythmia detection. The proposed model had flexible input length and halved parameter amount that reduced computation in real-time processing by 90% as compared to the conventional CNN model. The ATN-CN model achieved an accuracy of 81.2%. Vafaie et al. [135] proposed a heart disease prediction model through ECG signal classification using genetic-fuzzy system. The proposed fuzzy classifier method achieved an accuracy of 93.34%. Furthermore, with the application of genetic algorithm, the accuracy was enhanced up to 98.67%. Sahoo et al. [136] proposed a method for the detection of QRS complex features through multiresolution wavelet transform for the classification of four types of ECG beats. Features were extracted through principal component analysis (PCA). NN and SVM were used for the classification. The proposed system achieved an accuracy of 96.67% for NN and 98.39% for SVM.

RETRACTED

Dohare et al. [137] developed a system for myocardial infraction detection in 12-lead ECG through SVM. The average beat of ECG was determined through the 12-lead ECG by using four clinical features such as ST-T complex interval, QT interval, *P* duration, and QRS duration. The principal component analysis (PCA) was used in the proposed method for the reduction of feature dimension. The dataset used for the validation of the proposed method was collected from Physikalisch-Technische Bundesanstalt (PTB) database. SVM was employed for the classification. The proposed MI detection method achieved an accuracy with specificity and sensitivity of 98.33%, 100%, and 96.66%, respectively.

An artificial intelligent- (AI-) enabled electrocardiograph (ECG) based on CNN for the detection of electrocardiography signature of atrial fibrillation was proposed by Attia et al. [138]. The patients data was collected from the Mayco Clinic ECG laboratory consisting of 180922 patient records with 649931 normal subjects. The receiver operating characteristic (ROC) curve was used to validate the results of the proposed method. The proposed model obtained an accuracy, specificity, and sensitivity of 87%, 79%, and 79.5%, respectively. Melgare et al. [139] explored ML approaches for the detection of electrocardiography fragment activity. For this reason, four different datasets were utilized along with three additional databases. For the classification problem, SVM, decision tree (DT), and Gaussian Naive Bayes (NB) were used for deep analysis of the selected datasets. The best results obtained for the fragmented dataset were 94% sensitivity, 88% specificity, 89% positive predictive value, 93% negative predictive value, and 91% accuracy when using SVM with Gaussian kernel.

RETRACTED

Feng et al. [140] proposed a model for myocardial infarction classification through CNN and Recurrent_NN. A raw data was processed with the proposed algorithm to extract heart beat segments. After feature extraction, CNN and LSTM were deployed for ECG classification. The dataset used for validating the proposed model was collected from Physikalisch-Technische Bundesanstalt (PTB). The proposed algorithm reported an accuracy, sensitivity, and specificity of 95.4%, 98.2%, and 86.5%, respectively. Kumar et al. [142] proposed a technique for automated diagnosis of myocardial infarction ECG signals based on the sample entropy in flexible analytic wavelet transform framework (FAWT). The FAWT model was implemented on every ECG beat which decomposed the ECG beats into the subband signal. Subband signals were used for computing the sample entropy (Sent) that was fed into the random forest, BRNN, and LS-SVM for classification. The highest accuracy of 99.31% was achieved through the LS-SVM.

Yin et al. [143] proposed a multidomain feature extraction method for arrhythmia classification. Dataset for the experiments was collected from the MIT-BIH arrhythmia database. 1-fold crossvalidation scheme was selected for performance evaluation of the proposed method and genetic algorithm used for the optimized selection of parameters. The average accuracy of 99.70% with sensitivity and specificity of 99.68% and 99.96%, respectively, was reported through the proposed method (SVM-RBF). Li and Zhou [152] proposed a method for ECG classification based on wavelet packet entropy and random forests. The dataset used in this study was collected from the MIT-BIH arrhythmia database. The proposed method used WPE + RR for feature extraction and random forest (RF) for classification and for which an accuracy of 94.61% was reported. Yang et al. [151] proposed a method for automatic recognition of arrhythmia using principal component analysis network and linear SVM. The principal component analysis network (PCANet) was used for the extraction of features from ECG signals while SVM was deployed for classification. For the experiment, MIT-BIH arrhythmia database was used to validate the effectiveness of the proposed model which achieved an accuracy of 97.94%.  Figure 9 provide the overview of various ML techniques performance based on ECG modality.

RETRACTED

## 4. State-of-the-Art Work

Ricciardi et al. [51] presented a tree-based ML method based on radiodensitometeric distribution for assessing the cardiovascular risks through mid-thigh CT image. The dataset was collected from AGES-I and AGES-II for the experimental purpose. The proposed method tested against the CHD, CVD, and CHF. The proposed method based on logistic regression and tree-based ML model achieved the accuracy for CHD (AUCROC: 0.936), CVD (AUCROC: 0.914), and CHF (AUCROC: 0.994). Butun et al. [52] developed a deep capsule network for the detection of CAD using ECG signals. The capsule network was designed through deep learning-based methods. The proposed method was given as 1D-CADCapsNet. The dataset was obtained from Physionet databases for the experiments. The accuracy reported by the 1D-CADCapsNet was 99.44%.

Ramachandran et al. [53] proposed a computerized diagnostic system for CVD based on photoplethysmography signals. The proposed system extracted the features from photoplethysmography through singular value decomposition (SVD), statistical features, and wavelets while Softmax Discriminant Classifier (SDC) and Gaussian mixture model classifier (GMM) were used for classification. The newly proposed system obtained an accuracy of 97.88%. Dataset used for the experiments was obtained from IEEE TMBE pulse oximeter dataset to evaluate the performance of the proposed computerized diagnostic system. Ghiasi et al. [54] proposed a decision tree-based diagnosis of CAD model named as CART. The newly designed CART model obtained the accuracy of 100% on Z-Alizadeh Sani CAD dataset.

Gjoreski et al. [56] proposed a deep learning-based method for the detection of chronic heart failure using heart sound. The dataset used in this study for experiments consisted of recordings from 947 subjects from six publicly available datasets. The newly proposed system achieved an accuracy of 93.2%. Hussain et al. [57] proposed a novel CHF based on multimodal extracting features and ML approaches. The RR interval time series data was used for experiments that were obtained from the Physionet databases. The highest accuracy of 97% was achieved by SVM linear kernel. Aouabed et al. [58] developed an ensemble model for early detection of CAD. The ensemble model is based on four different kernel functions (linear, polynomial, radial basis, and sigmoid). To analyze the performance of the proposed model, an online dataset from UCI repository was obtained. Genetic algorithm was employed for feature extraction. The proposed model achieved an accuracy of 98.34%. Liu et al. [59] proposed a multiscale convolutional neural network for coronary artery fibrous plaque detection. The coronary OCT images were collected from Peking Union Medical College Hospital, China, for experiments purpose. The proposed method obtained an accuracy of 94.12%. Moreover, the summary of state-of-the-art proposed models is reported in Table 2.

RETRACTED

## 5. Discussion

Herein, we scrutinized the top ten research articles from each modality based on accuracy and performance that were achieved on various datasets. Furthermore, a comparison of modality-based ML techniques is depicted in Figure 10, where modality-based ML models are ranked according to accuracy and number of samples used in the dataset. It can also be observed from Figure 10 that ML techniques based on ECG modality have better accuracy and performance as compared to clinical feature-based data modality. Furthermore, image modality has shown less accuracy in comparison to ECG and clinical feature-based data modality. Another factor that can be observed from Figure 10 is that clinical feature-based data modality and image modality-based ML techniques lose accuracy and performance when the number of samples or subjects were huge in the dataset, whereas ECG modality-based ML models performed well in case of huge or small number of samples in the datasets.

One of the key factor for an ML model to obtain the best performance is based on the nature of data that exists in the dataset. As we have observed, the three modalities used diverse datasets that means nature of data varies for each such as ECG signals, images, and medical reports data. Therefore, ECG modality-based ML models used signal data and obtained higher performance and accuracy as compared to other modalities for prediction and detection of the HF and CAD.

Feature selection/extraction is also an important part of ML-based models where we select the most appropriate feature from the feature space. The feature space is reduced by eliminating features from the feature space which helped to improve the performance and accuracy of ML models. Feature selection process differs from feature extraction in that, in the features selection process, only those features are selected from the feature vector that heavily contribute to achieving a better accuracy, while in the feature extraction process, new features are produced from the features space which increases the accuracy of the proposed ML models. Therefore, feature processing is an important part in ML models that not only does contribute to achieve higher accuracy but also reduces the model's computational cost. For example, in the ECG modality, features are extracted from the ECG signals through sampling of the signals. The most widely used methods for extracting features from the ECG signals are QR wave and R-R interval.

RETRACTED

Performance evaluation of the ML model is another key factor of ML pipeline. Numerous types of performance metrics are utilized to measure the performance of ML models, e.g., F1 score, area under the curve (AUC), ROC, Matthews correlation coefficient (MCC), specificity, sensitivity, and accuracy [153]. Another important factor is validation methods. Different validation methods, namely, train-test holdout validation, *k*-fold crossvalidation, and leave-one-out (LOO) crossvalidation methods have been used by different researchers. The ML-based model for automated diagnosis of HF and CAD detection mostly used *k*-fold crossvalidation metric for the evaluation of the newly developed model. The modalities (Tables 3–5) also show that *k*-fold crossvalidation method has been widely used by the researchers, while the performance of ML models with respect to modality can be seen from Figure 11 where SVM, RF, and DNN models have obtained higher accuracy as compared to the other ML models.

### 5.1. Limitations in the Previously Developed Methods

ML algorithms are applied to various problems in different application domains. However, they suffer from some limitations which make them imperfect for every problem. In the area of clinical support systems, most ML methods for automated diagnosis of HF, CAD, and CHF belong to the supervised learning category. Since supervised learning has some limitations, automated diagnosis systems also suffer from, if not all but some of these limitations. In this section, we address these limitations of ML-based methods

- Supervised ML models requisite training on the dataset; however, training on large amount of data is complex and time consuming task
- ML models may suffer from the data overfit problem. As discussed above, *k*-fold crossvalidation method has been widely utilized by many researchers for evaluating the performance of their developed diagnostic system. However, it may result in overfitted or highly biased results due to data leakage
- In recent years, deep learning technology has shown state-of-the-art performance on heart disease detection problem. However, the deep learning technology requires huge amount of data for model training which is a costly and difficult job
- Time complexity is another issue in automated detection of heart disease based on ML approaches. ML model can predict only after they have been trained on the training data which requires processing time. Moreover, ML models have many parameters, which needs to be tuned manually in case of supervised learning. Therefore, a lot of time is required to fine tune the hyper parameters of the ML model for achieving better performance
- Another drawback in many previously proposed methods and reported results is the biased comparative study in many papers, for example, comparing results of two studies which have used different validation methods (holdout and crossvalidation) or different evaluation metrics. For an unbaised comparison, it is important to use same dataset with same validation scheme and evaluation metrics

RETRACTED

### 5.2. Future Research Directions

Several ML models have been proposed for the prediction of CAD and HF in the past few years; however, there are some areas that still need to be explored by researchers and professionals. In this section, we have addressed the potential research areas and directions for further improvement in ML methods for CAD detection. Through this study, we conclude that there are three key factors that participate for efficient detection of the CAD and HF.

Firstly, data is very significant in case of ML-based automated detection of heart disease, especially, when deep learning models are brought into account. However, many of the publicly available datasets are small sized. Hence, future studies focus should be on collection of the large amount of datasets.

Secondly, as discussed above, *k*-fold crossvalidation-based model performance gives biased performance owing to data leakage. Hence, in future studies, in order to develop models that would show better generalization performance, an independent dataset should be used. After development of the model using crossvalidation, the developed model generalization capabilities should be blind tested on the independent dataset. Such type of generalized models would be of great help and could be deployed in hospitals for real time diagnosis.

Thirdly, ML is an emerging field; therefore, there are still open challenges for development of novel methods that will provide efficient performance.

Fourth, recently on many other disease detection problems, multimodal processing has provided reliable and efficient results. Hence, in future, researchers should exploit multimodal approaches for a better heart disease detection.

## 6. Conclusion

Unlike previous studies, in this study, we scrutinized various ML approaches for the development of automated diagnostic systems for heart disease detection based on different kinds of modalities (clinical features-based data, imaging, and ECG). Research articles were collected from various databases published between 1995 and 2021. Based on different data modalities, the previously proposed studies were critically analyzed and systematically organized. Moreover, in this study, we also pointed out the limitations and loop holes in the previously proposed methods for automated heart disease detection. Finally, to mitigate the problems present in previously developed methods and to provide better heart disease detection, some future directions were discussed for onward research in the domain of automated heart disease detection based on ML. We hope that this review will be helpful to those who intend to work in the domain of automated heart disease detection.

RETRACTED

## Figures and Tables

**Figure 1:** Anatomy of the heart [6].

**Figure 2:** Types of heart diseases.

**Figure 3:** Different modalities used for automated heart failure diagnosis.

**Figure 4:** Overview of ML-based diagnostic system.

**Figure 5:** Selected research articles published from 1996 to 2021 as shown in Figure 5(a). The topic has gradually attracted the attention of researchers with the passage of time. In recent years, the topic got a peak attraction from researchers as a lot of articles have been published in the past few years, while Figure 5(b) depicts the comparison of published articles with respect to the modality.

**Figure 6:** Demonstrates the number of samples and features in each dataset. *X*-axis of the graph represents the dataset ID while the *Y*-axis displays the number of samples and number of features. Blue bar in the figure depicts number of sample, and the orange line denotes number of features.

**Figure 7:** Performance of clinical feature-based data modality based on ML models is depicts from this figure. The performance of each ML model is measured in term of accuracy along with number of samples in the dataset.

**Figure 8:** Performance of ML models based on image modality is depicted in this figure. The performance of each ML model is measured in term of accuracy along with number of samples in the dataset.

**Figure 9:** Performance of ECG modality-based ML models is depicted in this figure. The performance of each ML model is measured in term of accuracy along with number of samples in the dataset.

**Figure 10:** Performance analysis of ML techniques based on datasets for automated diagnosis of heart failure. This figure shows the highest accuracy achieved by the clinical feature-based data modality-based methods while average accuracy of ECG modality-based methods is higher. As the number of samples in dataset is increased, the performance of the clinical feature-based data modality reduces. The image modality has shown lower performance as compared to the other two modalities.

**Figure 11:** The performance of ML models with respect to modality can be seen in this figure. SVM, RF, and DNN models have obtained higher accuracy as compared to the other ML models. Modalities of the ML models can also be seen in this figure.

RETRACTED

**Table 1:** Summary of dataset properties.

Dataset_ID^a^	Dataset	Total samples^b^	Features^c^
01	Cleveland (UCI), heart disease dataset	303	76 raw features, 14 prominent features
02	StatLog heart disease dataset (UCI)	150, (healthy: 150, patient: 120)	13 distinct features
03	CHF database (chf2db)	136, (healthy: 46, patient: 90)	12 distinct features
04	MIT-BIH Normal Sinus Rhythm (NSR) database	54, (male: 30, female: 24)	Sampling rate: 128 samples per second
05	Congestive heart failure database (BIDMC-CHF)	15, (male: 11, female: 4)	Sampling rate: 500 samples per second
06	Fantasia database (FD)	18, (male: 5, female: 13)	Sampling rate: 128 samples per second
07	Congestive Heart Failure RR Interval Database (CHF-RR)	29	Sampling rate: 500 samples per second
08	Normal Sinus Rhythm RR Interval Database (NSR-RR)	40	Sampling rate: 500 samples per second
09	Cleaveland(UCI), Hungarian heart disease dataset	590	76 features
10	mARSupio database, Italy	14616, (patients: 347)	572 features
11	NHANES CVD dataset	4434	23-65 features
12	MIMIC-II clinical database	8059	32 features
13	Z-Alizadeh Sani dataset	303	54 features
14	Heart disease dataset, Andhra Pradesh, India	N/A	14 features
15	Physionet databases	40, (male: 20, female:20)	95300 segmented ECG
16	MITDB database, Physionet	47	22 features
17	China Kadoorie Biobank (CKB)	520000	86 features
18	MIT-BIR arrhythmia database	47	Sampling rate of 360 Hz
19	MIT/Beth Israel hospital (BIH), arrhythmia database	4,000 ambulatory ECGs	360 samples per second
20	PTB diagnostic ECG database	52 healthy, 7 HCM, 8 DCM, and 148 MI subjects	Sampled at 1,000 Hz, 250 samples per second
21	Physikalisch-Technische Bundesanstalt diagnostic, ECG database	200 (patients: 148, healthy: 52)	Sampling rate of 1000 Hz
22	1st China Physio-logical Signal Challenge	6877	Sampled at 500 Hz
23	Mayo Clinic ECG laboratory	180922, (patients: 116061, healthy: 64931)	Sampling 1500 Hz
24	Subrogated fragmented database (Sfrag-DB) + subrogated wide-fragmented database (SWfrag-DB) + fragmented database (FHCM-DB) + fibrosis database (HCM-DB)	616 records	Sampling rate: 500 Hz
25	Collected at the University of Pennsylvania	209	20 features
26	MICCAI 2017 challenge on Automated Cardiac Diagnosis	100	567 features, 13 optimal features
27	STACOM 2015 challenge	200	11 features
28	St.Francis Heart Hospital in Roslyn, New York	200	3 feature
29	Nuclear Medicine Department	288	10 features
30	Cedars-Sinai Medical Center, Los Angeles, CA	713	13 features
31	MCG data	800	2 features
32	Hospital Fernando Fonseca dataset	496	80 features
33	Siemens Somatom sensation	137	N/
34	ACS dataset (Mersin University Research and Training Hospital)	228	6 features
35	University Hospital Arnau de Vilanova, Lleida, Spain	56	Image resolution: 8.5 pixels per mm
36	Sutter Palo Alto Medical Foundation	58652000	2 attribute
37	LIDC-IDRI public dataset	802	NoGT transformation
38	SunnyBrook Cardiac Data (SCD)	45 (male: 32 and female: 13)	Sampling: 30 frames per second
39	NSTEACS	2302 patients	N/A
40	Hospital Universiti Kebangsaan Malaysia	10	N/A
41	Department of Medicine, University of Alabama at Birmingham	109	9 features
42	UK Biobank	9135867	N/A
43	SPECT	135	30 Fourier components
44	Ham-mersmith Hospitals	1093 subjects	N/A
45	Cohn-Kanade dataset (CK+)	400	N/A
46	Sacred Heart Medical Center, Eugene	215	N/A
47	Sacred Heart Medical Center	2619	50 features
48	AGES-I Dataset	628 (male: 419, female: 209)	11 Radiodensitometric features
49	Clinical Research Centre of Medical University of Bialystok, Poland	67	63 features
50	Sugam Multispecialty Hospital, India	507 patients (35 to 90 years of age)	22 features
51	Germany	15510 observations	N/A
52	Italian Local Health Authority (ASL)	2722	06 features
53	ML repository	3000	13 features
54	USA	1000	15 echocardiographic variables
55	USA	340	15 echocardiographic variables
56	Faisalabad Institute of Cardiology and at the Allied Hospital in Faisalabad (Punjab, Pakistan)	299	13 features

^a^Dataset_ID is a reference number used for the identification of the dataset. ^b^Total samples represent the total number of records in a dataset. ^c^Feature represents the total number of features a dataset consist.

RETRACTED

**Table 2:** Summary of state-of-the-art research articles.

P_ID	Author	Technique	Data	Feature selection	Data sampling	Conclusion
PI_106	Ricciardi et al.,(2020) [51]	Logistic regression + tree-based ML	AGES-I dataset + AGES-II dataset	Nonlinear trimodal regression analysis (NTRA) + RF	*k*-fold crossvalidation *k* = 12	CVD (AUC: 91.4%) CHD (AUC: 93.6%) CHF (AUC: 99.4%)
PI_107	Butun et.al. (2020) [52]	Capsule networks (DNN)	Physionet database	Layer of CNN	Crossvalidation, 5-fold	Accuracy: 99.44%
PI_108	Ramachandran et al., (2020) [53]	Softmax discriminant classifier (SDC) and Gaussian mixture model classifier (GMM)	IEEE TMBE pulse oximeter dataset	Singular value decomposition (SVD)	*F*-measure	Accuracy: 97.88%
PI_109	Ghiasi et al. (2020) [54]	Decision tree	Z-Alizadeh Sani CAD dataset	Classification and regression tree (CART)	Crossvalidation,10-fold	Accuracy: 100%
PI_110	Joloudari et al. (2020) [55]	RT + SVM + C5.0	Z-Alizadeh Sani dataset	Random trees	Crossvalidation, 10-fold	Accuracy: 91.47%
PI_111	Ali et al. (2019) [42]	*L*_1_-regularized-linear-SVM stacked with nonlinear SVM	Cleveland (UCI), heart disease dataset	*L*_1_-regularized-linear-SVM	Matthews relation coefficient (MCC)	Accuracy: 92.22%
PI_112	Ali et al.,(2020) [43]	Mutual information based feature selection and deep neural network	Cleveland (UCI), heart disease dataset	Mutual information	Matthews relation coefficient (MCC)	Accuracy: 93.33%
PI_113	Gjoreski et al. (2020) [56]	Fully connected neural network (FCNN)	947 subjects	openSMILE feature extraction tool	Crossvalidation 10-fold	Accuracy: 93.2%
PI_114	Hussain et al. (2020) [57]	DT + SVM + KNN	Physionet databases	Multimodal features	Crossvalidation 10-fold	Accuracy: 97% (SVM)
PI_115	Aouabed et al. (2019) [58]	Nested ensemble (NE) model	Cleveland (UCI), heart disease dataset	GA	Crossvalidation 10-fold	Accuracy: 98.34%
PI_116	Liu et al. (2020) [59]	Multiscale convolutional neural networks (CNN)	1000 OCT images	Layers of CNN	Matthews relation coefficient (MCC)	Accuracy: 94.12%

RETRACTED

**Table 3:** Summary of clinical features-based data modality articles.

P_ID	Author	Technique	Data	Feature selection	Data-sampling	Conclusion
PI_01	Verma et al. (2016) [40]	FURIA + MLR+ clustering + MLP	Cleveland heart disease dataset, IGMC data	CFS + PSO	*k*-fold crossvalidation k =10	Accuracy: 90.28% Accuracy: 88.4%
PI_02	Shah et al. (2017) [41]	Radial basis function (RBF) kernel-based SVM	Cleveland heart disease dataset, 303 instances	PPCA+PA	*k*-fold crossvalidation *k* =10	Accuracy: 91.30% Sensitivity: 100%
PI_03	Dwivedi (2018) [44]	LR + KNN + ANN + NB + classification tree + vector machines (SVM)	StatLog heart disease dataset	N/A	*k*-fold crossvalidation k =10	Accuracy: 85% Sensitivity: 81% Specificity: 89%
PI_04	Haq et al. (2018) [60]	Logistic regression (LR) + KNN + ANN + NB + DT + SVM	Cleveland heart disease dataset, 303 instances	Relief + mRMR + LASSO	*k*-fold crossvalidation *k* =10	Accuracy: 89% Sensitivity: 96% Specificity: 98%
PI_05	Guidi et al. (2014) [45]	NN + SVM + fuzzy-genetic + regression tree + random forest	Cardiology Department at the St. Maria Nuova Hospital in Florence, Italy Records, 90 patients	N/A	*k*-fold crossvalidation *k* =10	Prediction accuracy: NN: 84.73%, SVM: 85.2%, FG: 85.9%, CART: 87.6%, RF: 85.6%
PI_06	Pawlovsky (2018) [46]	An ensemble based on distances for a kNN (*k* nearest neighbor)	Cleveland heart disease dataset, 303 instances	Distances(Mahalanobis) + voting scheme using weights	*k*-fold crossvalidation *k* =10	Accuracy: 84.83%
PI_07	Yu and Lee (2012) [47]	SVM+ bispectral analysis	CHF database (chf2db), Physionet database (nsr2db)	Bispectrum-related features + GA	*K*-fold crossvalidation *k* =10	Accuracy: 98.79%
PI_08	Wang et al. (2019) [48]	DNN + ensemble learning method	BIDMC-CHF, NSR-RR	Time, frequency domain, nonlinear features	Blindfold validation	Accuracy: 99.96%
PI_09	Methaila et al. (2014) [49]	NN + NB + DT + apriori (algorithm + MAFIA algorithm)	Cleveland heart disease dataset, 303 instances	Significance weightage calculation	Crossvalidation	Accuracy: 99.62% (DT)
PI_10	jan et al. (2018) [50]	Ensemble model + NB + ANN + weight+ random forest + SVM	Cleveland heart disease Hungarian dataset, 590 instances	N/A	*K*-fold crossvalidation (*k* = 10)	NB: 93.22%accuracy ANN: 94.91%, accuracy SVM: 98.13%, accuracy LR: 93.22%, accuracy
PI_11	ali et al.(2019) [42]	Optimized stacked support vector machines	Cleveland heart disease dataset, 303 instances	SVM with kernels including linear + RBF.	Matthews correlation coefficient (MCC)	Accuracy: 92.22%
PI_12	Pecchia et al. (2010) [61]	CART	CHF RR interval database	Short-term HRV analysis	MCC + ROC	Accuracy: 96.39%,
PI_13	Kurnar (2012) [62]	ANN + fuzzy logic	Cleveland heart disease dataset, 303 instances	Fuzzy resolution	Matthews correlation coefficient (MCC)	Accuracy: 91.83%
PI_14	Kurnar (2012) [62]	LR + RF + NB + GB + SVM	Cleveland, Hungarian, Switzerland	Data cleaning	Confusion matrix	Accuracy: 86%
PI_15	Panicacci et al. (2019) [63]	RF+ MACRO +SMOTE28 S	mARSupio database, Italy. 14616 subjects, 347 patient	N/A	F1-score, F2-score	Accuracy: 98.74%
PI_16	Beulah et al. (2019) [64]	Majority vote with NB, BN, RF, and MP	Cleveland heart disease dataset, 303 instances	Bagging, MV, stacking, boosting	F1-score, F2-score	Accuracy: 85.48%
PI_17	Zikos et al. (2019) [65]	Conditional probability +Bayesian	Medicare and Medicaid services CMS, 564,875 records	Clinical Classification Software (CSS)	N/A	Mortality rate: 2.61%
PI_18	Daset et al. (2009) [5]	Neural networks ensembles	Cleveland heart disease dataset, 303 instances	SAS base software 9.1.3 for diagnosing	MCC + ROC	Accuracy: 89.01%
PI_19	Mohan et al. (2019) [66]	Hybrid random forest with a linear model	Cleveland heart disease dataset, 303 instances	NB, GLM, LR, DL, DT, RF, GBT, and SVM	Confusion matrix	Accuracy: 88.4% Sensitivity: 90.8% Sensitivity: 82.6%
PI_20	Kahramanli and Allahverdi (2008) [67]	ANN + FNN	Cleveland heart disease dataset, 303 instances	N/A	*k*-fold crossvalidation	Accuracy: 86.8%
PI_21	Maji and Arora (2018) [68]	Decision tree+C4.5 + ANN	UCI, dataset with 13 attributes and 270 instances	Pruning	*k*-fold crossvalidation	Accuracy: 78.14%
PI_22	Polat et al. (2005) [69]	Fuzzy weighted + AI	Cleveland heart disease dataset, 303 instances	Fuzzy weighted preprocessing	*k*-fold crossvalidation	Accuracy: 96.30%
PI_23	Ster and Dobnikar (1996) [70]	Neural networks	CAD:263 subjects, UCI: 297	N/A	*k*-fold crossvalidation.	HD accuracy: 84.5% CAD accuracy: 59.7%
PI_24	Chen et al. (2017) [71]	Deep learning with RR intervals	72 healthy persons and 44 CHF patients	Autoencoder	*k*-fold crossvalidation	Accuracy: 72.41
PI_25	Purushottam and Sharma (2015) [72]	Decision trees	Cleveland heart disease dataset, 303 instances	C4.5	Confusion matrix	Accuracy: 87%
PI_26	Rajliwall et al. (2018) [73]	ML-based models for cardiovascular risk prediction	NHANES dataset + Framingham heart study dataset	C4.5	Fivefold crossvalidation	Accuracy (RF): 98.5%
PI_27	Samuel et al. (2017) [74]	ANN and Fuzzy_AHP	Cleveland heart disease dataset, 303 instances	Fuzzy_AHP	ROC	Accuracy: 91.10%
PI_28	Venkatalakshmi and Shivsankar (2014) [75]	Decision tree + naive Bayes (NB)	Cleveland heart disease dataset, 303 instances	Weka tool	Confusion matrix	NB: 85.03%accuracy
DT: 84.01%accuracy						
PI_29	Maio et al. (2017) [76]	Random survival forest	MIMIC II clinical database, 8059	N/A	OOB, C-statistics	Accuracy: 82.01%
PI_30	Arabasadi et al. (2017) [34]	Hybrid neural network-genetic algorithm	Z-Alizadeh Sani dataset	Genetic algorithm	10-fold crossvalidation	Accuracy: 93.85%
PI_31	Abdar et al. (2017) [77]	N2Genetic optimizer + N2Genetic-nuSVM	Z-Alizadeh Sani dataset	GA + PSO	Crossvalidation 10-fold + F1-score	Accuracy: 93.08% *F*-score: 91.51%
PI_32	Mezzatesta et.al. (2019) [78]	LR + KNN + CART + NB + SVM	HEMO clinical trial + IFC-CNR, Italy	Scaling techniques	Crossvalidation *K*-fold	LR: 80%, SVM: 80%
PI_33	Lakshmi et al. (2016) [79]	NB classifier + SVM	Cleveland heart dataset	Reprocessing	ROC	NB: 84.87%, accuracy SVM: 93.08%
PI_34	Bashir et al. (2019) [80]	DT + NB + LR + SVM	Cleveland heart disease dataset, 303 instances	MRMR	5-fold crossvalidation	Accuracy: 84.85%
PI_35	javeed et al. (2019) [81]	RSA + ORFA	Cleveland heart dataset	Hybrid Feature Subset	MCC	Accuracy: 93.33%

RETRACTED

**Table 4:** Summary of image modality based research articles.

P_ID	Author	Technique	Data	Feature selection	Data sampling	Conclusion
PI_36	Nirschl et al. (2018) [83]	CNN+ whole-slide images of H&E tissue	209 patients	WND-CHARM	*k*-fold crossvalidation	Accuracy: 97.4%
PI_37	Cetin et al. (2017) [84]	Radiomic approach + cardiac cine-MRI+ SVM	MICCAI 2017 challenge on automated cardiac diagnosis	Sequential forward feature selection (SFFS)	Crossvalidation	Accuracy: 98%
PI_38	Bai et al. (2016) [85]	SVM	STACOM 2015 dataset	ED + ES phases + PCA	*k*-fold crossvalidation	Accuracy: 97.5%
PI_39	Qazi et al. (2007) [86]	SLFD	200 cases	LFD	ROC + *k*-fold crossvalidation	Accuracy: 89.1%
PI_40	Sajn and Kukar (2011) [87]	Image processing + ML	288 patients	PCA	ROC + *k*-fold crossvalidation	Accuracy: 81.3%
PI_41	R.Arsanjani et al.,(2015) [88]	Myocardial perfusion SPECT + ML	Cedars-Sinai Medical Center	LogitBoost	ROC + *k*-fold crossvalidation	Accuracy: 81%
PI_42	Arsanjani et al. (2013) [89]	SPECT for detection of CVD	Cedars-Sinai Medical Center	LogitBoost	ROC + *k*-fold crossvalidation	Accuracy: 87.2%
UPI_43	Udovychenko et al. (2015) [90]	*k*-NN binary classification of heart failures	MCG data	Variance, kurtosis, and skewness	MMC	Accuracy: 80-88%
PI_44	Carneiro and Nascimento (2013) [91]	Multiple dynamic models and deep learning architectures	Hospital Fernando Fonseca dataset, 496 images	PCA	HMD, AV, MAD, AVP	d_HMD: 83%accuracy d_AV: 91%accuracy d_MAD: 94%accuracy d_AVP: 83%accuracy.
PI_45	Zheng et al. (2008) [92]	3-D cardiac CT volumes using marginal space learning	Siemens Somatom Sensation	Steerable features	*k*-fold crossvalidation	Mean error: 2.3%
PI_46	Berikol et al. (2016) [93]	SVM	Mersin University Research	N/A	*k*-fold crossvalidation	Accuracy: 99.13%
PI_47	Lekadir et al. (2016) [94]	Plaque CNN architecture	Arnau de Vilanova	Deep learning CNN	*k*-fold crossvalidation	Accuracy: 80%
PI_48	Sundaresan et al. (2017) [95]	Fully convolutional neural networks (FCN)	C.Ioannou	Rectified linear units (ReLUs)	ROC	Classification error rate: 23.48%
PI_49	Choi et al. (2016) [96]	Recurrent neural network	Sutter Palo Alto Medical Foundation	Gated recurrent unit GRU	*k*-fold crossvalidation *k* =6	Accuracy: 88.3%
PI_50	Toth et al. (2018) [97]	Convolutional neural networks	LIDC-IDRI public dataset	(ReLU)	Qualitatively + quantitatively	Error rate: 2.92%
PI_51	Maraci et al. (2017) [98]	Analysis of linear ultrasound videos to detect fetal presentation and heartbeat	Dataset of 323 predefined free-hand videos	PCA	*k*-fold crossvalidation *k* = 5	Accuracy: 93.1%
PI_52	Kurgan et al. (2001) [99]	Automated cardic SPECT diagnosis	Database of features(DF)	CLIP algorithm	Qualitative and Quantitative test	Accuracy: 83.08%
PI_53	Moreno et al. (2019) [100]	Multiscale motion for cardiac disease prediction	SPECT images dataset	RF + CLIP algorithm	F1-score + *k*-fold crossvalidation	Accuracy: 51.06% F1-score: 37.8%.
PI_54	Liu et al. (2016) [101]	ML prediction for cardiovascular	NSTEACS	PCA + MCE	*k*-fold crossvalidation	Accuracy: 75%
PI_55	Shin et al. (2016) [102]	Deep convolutional neural networks for computer-aided detection	ImageNet dataset for CAD	CNN features of AlexNet pretrained + GoogleNet-RI	k-fold crossvalidation *k* = 5	Accuracy:95%
PI_56	Hisham et al. (2011) [103]	Grid independent technique	10 patients	Grid the images	Linear correlation	Accuracy:80%
PI_57	Allison et al. (2005) [104]	ANN	LAD model	Crossvalidation	Accuracy: 92%	
PI_58	Welikala et al. (2017) [105]	Automated arteriole and venule classification using deep learning	UK Biobank	RGB and HSI color spaces	Crossvalidation	Accuracy: 86.97%
PI_59	Curiale et al. (2017) [106]	Deep learning network in cardiac MRI	Sunnybrook Cardiac Dataset (SCD)	RGB and HSI color spaces.	Dice's coefficient	Accuracy: 90%
PI_60	Lindahl et al. (20197) [107]	Interpretation of myocardial SPECT perfusion images using ANN	Sunnybrook Cardiac Dataset (SCD)	Two-dimensional Fourier trans form technique	ROC + *k*-fold crossvalidation *k* = 2	Sensitivity: 54.4% Specificity: 70.5%
PI_61	Bai et al. (2015) [108]	Statistical parametric mapping(SPM) + linear model	Hammersmith Hospitals	PCA	Dice overlap metric + mean surface distance	LV_cavity:0.950 ± 0.024 Myocardium: 0.824 ± 0.062 RVcavity: 0.909 ± 0.03
PI_62	Moreno et al. (2019) [109]	Regional multiscale motion representation for cardiac disease prediction	Sunnybrook Cardiac Data (SCD)	Random Forest algorithm (RaF)	No. true positive over total of samples + F1-score	Accuracy: 77.83% F1-score:76.92%
PI_63	Gulsun et al. (2016) [110]	Coronary centerline extraction + CNN	CTA datasets	CNN	Up-to-first-error evaluation	Sensitivity: 97% Specificity = 90%
PI_64	Narula et al. (2016) [111]	Automate morphological and functional assessments in 2D echocardiography	77 ATH+ 62 HCM patients	Information gain (IG) algorithm	*K*-fold crossvalidation	Sensitivity: 96% Specificity = 77%
PI_65	Carneiro et al. (2011) [112]	Deep learning architectures and derivative-based search methods	Cohn-Kanade dataset (CK+)	PCA	ROC + HMD, HDF, MAD, MSSD	d_AVP: 95%
PI_66	Xu et al. (2012) [113]	Transient ischemic dilation for coronary artery disease in quantitative analysis	Nuclear Medicine Department, Sacred Heart Medical Center, Eugene	Mibi-Mibi TID	Standard deviation (SD)	Sensitivity: 76%
PI_67	Betancur et al. (2017) [114]	ML	Sacred Heart Medical Center	*k*−fold crossvalidation	Quantitative imaging analysis	Accuracy: 81%
PI_68	Coenen et al. (2018) [115]	ML + coronary computed tomographic	351 patients	ROC	ML-based CT-FFR model	Accuracy: 73%
PI_69	Wolterink et al. (2015) [116]	CNN	116 CT patients	*k*−-fold crossvalidation	ML-based CT-FFR model	Accuracy: 95%
PI_70	Nakazato et al. (2010) [117]	Perfusion imaging for detection of CAD	142 patients	N/A	*k*−-fold crossvalidation	Accuracy: 95%

RETRACTED

**Table 5:** Summary of ECG modality based research articles.

P_ID	Author	Technique	Data	Feature selection	Data sampling	Conclusion
PI_71	Zhao et al. (2019) [118]	HRV + PTTV + SVM	40 heart failure patients	RR + PTT	*k*-fold crossvalidation	Accuracy: 90%
PI_72	Sudarshan, et al. (2017) [119]	DTCWT-based methodology	BIDMC + rhythm (NSR) + fantasia	ROC + *t*-test	*k*-fold crossvalidation	Accuracy: 99.86%
PI_73	Acharya et al. (2017) [120]	CNN + ECG signal	Physionet databases	Single CNN structure	*k*-fold crossvalidation	Accuracy: 95.1%
PI_74	Chen et al. (2019) [121]	Two-step predictive framework for ECG	MITDB + Physionet	Daubechies wavelet + PCA	*k*-fold crossvalidation	Accuracy: 96.26%
PI_75	Shen et al. (2016) [122]	Generative kernel density estimator	China Kadoorie biobank (CKB)	RR interval + P wave duration	*k*-fold crossvalidation	One-class: 75.6% Acc Four-class: 75.1% Acc
PI_76	Acharya et al. (2016) [123]	Automated diagnosis of serious arrhythmias	MIT-BIH A-fib + MIT-BIR arrhythmia	Approximate entropy	Confusion matrix	Accuracy: 96.3% %
PI_77	Mathews et al. (2018) [124]	Deep learning	MIT/Beth Israel Hospital (BIH)	Heartbeat interval features + RR intervals	MCC	Accuracy: 96.94% Sensitivity: 85.22%.
PI_78	Adam et al. (2018) [125]	DWT + nonlinear features	PTB Diagnostic ECG Database	SFS	10-fold crossvalidation	Accuracy: 99.27%
PI_79	Tan et al. (2018) [126]	Stacked convolutional + long short-term memory network	Physionet database	CNN	10-fold crossvalidation	Accuracy: 99.85%
PI_80	Sharma et al. (2018) [127]	Two-band optimal biorthogonal filter bank (FB)	Physikalisch-Technische ECG database	Fuzzy entropy + signal-fractal-dimension+ Renyi entropy	10-fold crossvalidation	Noisy data:99.62%, Acc Clean data: 99.74%, Acc
PI_81	Puceret et.al. (2018) [128]	Topological approach	MIT-BIH database	ADMT	10-fold crossvalidation	Accuracy: 92.73%
PI_82	Huang et.al. (2011) [129]	Vector cardiogram-based classification	PTB database from Physionet	FFS + BFS	10-fold crossvalidation	Accuracy: 96.96% Sensitivity: 99.89% Specificity: 92.51%
PI_83	Zhou et.al. (2018) [130]	Premature ventricular contraction + RNN	MIT-BIH arrhythmia database	Long short-term memory (LSTM)	Detection indexes	Accuracy: 96-99% Sensitivity: 99-100% Specificity: 94-96%
PI_84	U.Satija et al.,(2018) [131]	ECG signal quality assessment algorithms	MIT-BIH arrhythmia database	CEEMD + temporal features	10-fold crossvalidation	Accuracy: 98.80%
PI_85	Sudarshan et al. (2017) [119]	Dual tree complex wavelet transform	PhysioBank MIT-BIH NSR + fantasia + BIDMC CHF	Statistical features extracted from 2 seconds of ECG signals	10-fold crossvalidation	Accuracy: 99.86% Sensitivity: 99.78% Specificity: 99.94%
PI_86	Diker et al. (2019) [132]	Genetic algorithm wavelet kernel	Physikalisch-Technische Bundesanstalt diagnostic ECG database (PTBDB)	Discrete wavelet transform (DWT)	10-fold crossvalidation	Accuracy: 95% Sensitivity: 100% Specificity: 80%
PI_87	Acharya et al. (2017) [133]	Deep CNN	PTBDB	N/A	10-fold crossvalidation	Accuracy: 95.22% Sensitivity: 95.49%
PI_88	Yao et al. (2020) [134]	Attention-based time-incremental convolutional neural network (ATI-CNN)	1^*st*^ China Physiological Signal Challenge	CNN-LSTM, 1^st^ layer	Matthews correlation coefficient(MCC)	Accuracy: 81.2%
PI_89	Vafaie et al. (2014) [135]	Genetic-fuzzy + dynamical model of ECG signals	Physionet database	IF, THEN rules	N/A	Accuracy: 93.34%
PI_90	Sahoo et al. (2017) [136]	Multiresolution wavelet transform + ECG classification	MIT-BIH arrhythmia database	Principal component analysis (PCA)	10-fold crossvalidation	NN: 93.34% Acc SVM: 98.39% Acc
PI_91	Dohare et al. (2018) [137]	Myocardial infarction (MI) detection + SVM	Physikalisch-Technische Bundesanstalt (PTB)	Principal component analysis (PCA)	10-fold crossvalidation	Accuracy: 96.66% Sensitivity: 96.66% Specificity: 96.66%
PI_92	Attia et al. (2019) [138]	(AI)-enabled electrocardiograph (ECG) using a convolutional neural network	Mayo Clinic ECG laboratory	Non-linear ReLU	ROC	Accuracy: 87% Sensitivity: 79% Specificity: 79.5%
PI_93	Melgare et al. (2019) [139]	ML approach + electrocardiographic fragmented	Sfrag-DB + SWfrag-DB + FHCM-DB + HCM-DB	Statistics + PCA	Matthews correlation coefficient (MCC)	Accuracy: 90% Sensitivity: 94.1% Specificity: 87.5%
PI_94	Feng et al. (2019) [140]	CNN + RNN	PTB database	CNN and LSTM	10-fold crossvalidation	Accuracy: 95.4%
PI_95	Raka et.al. (2017) [141]	Time-based detection	SDDB + MIH-BIH database (NSRDB)	R-R interval duration	5-fold crossvalidation	Accuracy: 83.9%
PI_96	Kumar et al. (2017) [142]	ECG beat with flexible analytic wavelet transform (FAWT) + LS-SVM	ECG database from the Physiobank	Sample entropy (SEnt)	10-fold crossvalidation	Accuracy: 99.31%
PI_97	Yin et al. (2019) [143]	LS-SVM + multidomain electrocardiogram	MIT-BIH arrhythmia database	RR intevals, DWT, SampEn	10-fold crossvalidation	Accuracy: 99.31%
PI_98	Sahoo et al. (2017) [144]	SVM + NN	MITBIH arrhythmia database	Multiresolution wavelet transform	10-fold crossvalidation	Accuracy: 98.39%
PI_99	Masetic et al. (2016) [145]	Random forest	BIDMC CHF database (CHFDB) + NSRDB.	Autoregressive burg method	10-fold cross validation	Accuracy: 100%
PI_100	Isler and Kuntalp (2007) [146]	Classical HRV indices with wavelet entropy measures	MIT/BIH database	Genetic algorithm	Crossvalidation	Accuracy: 91.33% Sensitivity: 100%
PI_101	Bhurane et al. (2019) [147]	Frequency localized filter banks	NSRDB +BIDMC	Feature extraction	10-fold crossvalidation	Accuracy:99.66%
PI_102	Orhan (2013) [148]	Discretization method	NSRDB + BIDMC	EFiA-EWiT	10-fold crossvalidation	Accuracy: 99.33%
PI_103	Liao et al. (2015) [149]	SVM	CHFDB + MIT-BIH NSR database NSRDB	QRS wave	Ratio (ACC/SV)	Accuracy: 97.27%
PI_104	Yıldırım et.al. (2018) [150]	Deep CNN	MIT-BIH arrhythmia database	PCANet algorithm	Confusion matrix of	Accuracy: 95.20%
PI_105	Yang et al. (2018) [151]	LS-SVM + PCA	MIT-BIH database	PCANet algorithm	10-fold crossvalidation	Accuracy: 97.94%

RETRACTED

## Data Availability

The data that support the findings of this study are available upon request from the first author.
